# Correlation of matrix metalloproteinase 3 and matrix metalloproteinase 9 levels with non-motor symptoms in patients with Parkinson’s disease

**DOI:** 10.3389/fnagi.2022.889257

**Published:** 2022-08-22

**Authors:** Chuan Ze Liu, Da Shuai Guo, Jian Jun Ma, Lin Rui Dong, Qing Qing Chang, Hong Qi Yang, Ke Ke Liang, Xiao Huan Li, Da Wei Yang, Yong Yan Fan, Qi Gu, Si Yuan Chen, Dong Sheng Li

**Affiliations:** ^1^Department of Neurology, Henan University People’s Hospital, Zhengzhou, China; ^2^Department of Neurology, Henan Provincial People’s Hospital, Zhengzhou, China; ^3^Department of Neurology, Zhengzhou University People’s Hospital, Zhengzhou, China

**Keywords:** Parkinson’s disease, matrix metallopeptidase 3, matrix metallopeptidase 9, nonmotor symptom, cross-sectional study

## Abstract

**Objective:**

Matrix metalloproteinases (MMPs) are essential for tissue formation, neuronal network remodeling, and blood–brain barrier integrity. MMPs have been widely studied in acute brain diseases. However, the relationship with Parkinson’s disease (PD) remains unclear. The purpose of this study was to evaluate the serum MMP3 and MMP9 levels of PD patients and analyze their correlation with non-motor symptoms.

**Methods:**

In this cross-sectional study, we recruited 73 patients with idiopathic PD and 64 healthy volunteers. Serum MMP3 and MMP9 levels were measured by enzyme-linked immunosorbent assay (ELISA). Patients with PD were assessed for non-motor symptoms using the Non-motor Symptoms Scale (NMSS) and Parkinson’s disease sleep scale (PDSS) and Mini Mental State Examination (MMSE).

**Results:**

Serum MMP3 levels were significantly decreased in PD patients, predominantly those with early-stage PD, compared with controls [12.56 (9.30, 17.44) vs. 15.37 (11.33, 24.41) ng/ml; *P* = 0.004], and the serum MMP9 levels of PD patients were significantly higher than those of healthy controls [522 (419, 729) vs. 329 (229, 473) ng/ml; *P* < 0.001]. MMP3 levels were positively correlated with the NMSS total score (*r* = 0.271, *P* = 0.020) and the single-item scores for item six, assessing the gastrointestinal tract (*r* = 0.333, *P* = 0.004), and there was an inverse correlation between serum MMP3 levels and PDSS score (*r* = –0.246, *P* = 0.036); meanwhile, MMP9 levels were positively correlated with the NMSS total score (*r* = 0.234, *P* = 0.047), and higher serum MMP9 levels were detected in the cognitive dysfunction subgroup than in the cognitively intact subgroup [658 (504, 877) vs. 502 (397, 608) ng/ml, *P* = 0.008].

**Conclusion:**

The serum MMP3 level of PD patients (especially early-stage patients) was significantly lower than that of the healthy control group, and the MMP9 level was significantly higher than that of the healthy control group. MMP3 and MMP9 levels correlate with sleep disturbance and cognitive function in PD patients, respectively.

## Introduction

Parkinson’s disease (PD) is a chronic neurodegenerative disease characterized by the progressive loss of dopamine-producing neurons in the substantia nigra. Typical clinical symptoms include bradykinesia, resting tremor, and rigidity (Gao et al., 2003). PD is also associated with many non-motor symptoms, including cognitive decline, sleep disorders and depression, as well as gastrointestinal and genitourinary disorders (Schapira et al., 2006).

MMPs are a family of zinc-dependent endoproteases that play a variety of roles in tissue remodeling and degradation of various proteins in the extracellular matrix (ECM). MMPs promote cell proliferation, migration and differentiation and can play a role in apoptosis, angiogenesis, tissue repair and the immune response. The long-term role of matrix metalloproteinases (MMPs) in neurodegenerative diseases includes white matter damage in patients with vascular cognitive impairment, amyloid peptide degradation in Alzheimer’s disease, and dopaminergic neuronal apoptosis in PD (Rosenberg, 2009). In recent years, neuroinflammation has been considered an essential factor in the pathogenesis and development of PD (Hirsch and Hunot, 2009; Hirsch et al., 2012; Kaur et al., 2017), and MMPs are increasingly being found to be involved in the regulation of many common neuroinflammatory processes in neuropathology. Previous studies have shown that MMPs, as inflammatory mediators, participate in the activation of microglia and the production of superoxide, which ultimately leads to the degeneration of the substantia nigra and striatum and causes dopamine neuron death (Kim et al., 2007; Kim S. T. et al., 2010; Annese et al., 2015). Data from experimental studies have revealed that compared with healthy controls, MMP3 and MMP9 levels in postmortem brain tissue from patients with PD are increased (Lorenzl et al., 2002; Choi et al., 2008). In addition, in the MPTP mouse model of PD, ghrelin and exendin-4 have been shown to reduce the loss of DA neurons in the substantia nigra and striatum and the activation of microglia by inhibiting the expression of MMP3 (Kim et al., 2009; Moon et al., 2009), and reducing the expression of MMP9 may have the potential to treat PD (Lorenzl et al., 2004; Kim S. Y. et al., 2010; Lee et al., 2010; Broom et al., 2011). More importantly, MMP3 and MMP9 have been detected in the plasma (Lorenzl, 2003; Lorenzl et al., 2008; Horstmann et al., 2010; Tuna et al., 2018), serum (Liuzzi et al., 2002; Niebroj-Dobosz et al., 2010), and cerebrospinal fluid (Liuzzi et al., 2002; Adair et al., 2004; Horstmann et al., 2010; Niebroj-Dobosz et al., 2010; Bjerke et al., 2014) of patients with certain diseases, such as amyotrophic lateral sclerosis, Alzheimer’s disease, and leukodystrophy.

However, there is a dearth of data on the levels of MMPs in PD patients, and there are no previous studies exploring the potential relationship between serum MMP3 and MMP9 levels and the non-motor symptoms of PD. In this study, we aimed to assess serum MMP3 and MMP9 levels in PD patients with different clinical characteristics. As a secondary objective, we aimed to explore the correlation of MMP3 and MMP9 levels with motor and non-motor symptoms in PD patients.

## Materials and methods

### Participants

All participants were recruited from the Henan Provincial People’s Hospital. A total of 73 PD patients from the inpatient ward were consecutively recruited from September 2020 to December 2021. All patients were all assessed using the International Parkinson and Movement Disorder Society (MDS) Clinical Diagnostic Criteria for the clinical diagnosis of PD (Postuma et al., 2015). The exclusion criteria were as follows: (1) patients with acute cerebrovascular disease; (2) patients with acute or chronic infections in the last 3 months; (3) patients with autoimmune diseases such as rheumatoid arthritis; (4) patients with tumorous diseases such as glioma. Healthy age- and sex-matched volunteer controls were recruited at the same time from the health examination center. A total of 64 healthy volunteers participated in this study. None of the participants received any hormone therapy during the study period. All subjects were aware of the research content and provided written informed consent. The research protocol was approved by the Ethics Committee of Henan Provincial People’s Hospital of Medical Science.

### Clinical assessment

The demographic data and medical history of the included participants were recorded. The severity of motor symptoms was assessed using the Unified Parkinson’s Disease Rating Scale (UPDRS) Part III motor score (Gallagher et al., 2012) and Hoehn–Yahr (H-Y) stages (Goetz et al., 2004). According to the modified H-Y scale, we divided patients into two groups, with the early-stage PD corresponding to H-Y stages 1–2.5 and the advanced-stage PD corresponding to H-Y stages 3–5 (Goetz et al., 2004). Non-motor symptoms were assessed with the Non-motor Symptoms Scale (NMSS) (Chaudhuri et al., 2007) for PD, including total and single-item scores. Sleep disorders were assessed with the Parkinson’s disease sleep scale (PDSS). The PDSS is used to quantify all aspects of nocturnal sleep problems in PD, including overall quality of night’s sleep (item 1), sleep onset and maintenance insomnia (items 2 and 3), nocturnal restlessness (items 4 and 5), nocturnal psychosis (items 6 and 7), nocturia (items 8 and 9), nocturnal motor symptoms (items 10–13), sleep refreshment (item 14), and daytime dozing (item 15). The maximum score for each individual item is 10 points, with a maximum total score of 150 points. The lower the score is, the more pronounced the sleep disorder (Chaudhuri et al., 2002). A score of 90 or less indicates a sleep disorder (Porter et al., 2008). Cognition was examined by the Simple Mental State Examination (MMSE), adjusted for age and education level. Finally, the individual levodopa equivalent daily dose (LEDD) was calculated for each PD patient. All scale assessments were completed once during each patient’s “on” period.

### Blood sample collection

Peripheral blood was collected from each subject in test tubes without anticoagulant from 07:30 to 08:30 a.m. after an overnight fast and before breakfast. The sample was allowed to coagulate at room temperature for 30 min, the blood was centrifuged (1,000 × g, 15 min), and the serum was removed and stored at –80°C until measurement.

### Measurement of serum MMP3 and MMP9

Serum MMP3 levels were measured using an enzyme-linked immunosorbent assay (ELISA) kit (DMP300; R&D Systems, Minneapolis, MN, United States). The detection range of this kit is 0.2–10 ng/ml, the sensitivity is 0.045 ng/mL, and the intra- and interdetection variability ranges are 5.7∼6.4% and 7.0∼8.6%, respectively. Serum MMP9 levels were measured using an ELISA kit (DMP900; R&D Systems, Minneapolis, MN, United States). The detection range of the kit is 0.3–20 ng/mL, the sensitivity is 0.156 ng/mL, and the intra- and interdetection variability ranges are 1.9∼2.9% and 6.9∼7.9%, respectively. Biological replicates were analyzed on the same plate according to the manufacturer’s instructions.

### Statistical analysis

The normality of distributions was assessed using the *Shapiro–Wilk (SW)* normality test. Continuous data with a normal distribution are expressed as the mean ± standard deviation (SD). Data that did not conform to a normal distribution are expressed as median (25th–75th percentile). The normally distributed data of two groups were compared by independent sample Student’s *t* test. *One-way ANOVA* was used to compare data of multiple groups consistent with a normal distribution and homogeneity of variance, and a *post hoc least significant difference (LSD)* test was used to further compare the differences. Variables that did not conform to a normal distribution were evaluated by the *Mann–Whitney U*-test (two groups) or *Kruskal–Wallis (KW)* rank sum test (three or more groups). *Pearson* (or *Spearman*) correlation analysis was performed according to whether the variables are or are not normally distributed. The diagnostic sensitivity (Se) and specificity (Sp) values of biomarkers were assessed by receiver operating curve (ROC) analysis and cutoff point calculations. Statistical analysis was performed using SPSS version 21.0 (IBM Corporation, Armonk, NY, United States) and GraphPad Prism 8 (GraphPad Software, Inc., San Diego, CA, United States). A *P* < 0.05 was considered statistically significant.

## Results

### Clinical characteristics

Of the 137 study subjects, 73 PD patients (mean age 64.23 ± 8.95 years, 50.7% male, and 49.3% female) and 64 controls (mean age 62.50 ± 6.66 years, 48.4% male, and 51.6% female) were enrolled. In the PD group, the median duration of disease was 3 years. According to the levodopa equivalent conversion formula, the median LEDD was 400.0 mg, and the average score of the third part of the UPDRS was 28.88 (Table 1). There were no significant differences in sex or age between PD patients and healthy controls (*P* > 0.05).

**TABLE 1:** Clinical characteristics and serum MMP3 and MMP9 levels of participants in individual groups in the current study.

Characteristics	PD (*n* = 73)	Controls (*n* = 64)	*t*/χ^2^	*P*-value
Age, y	64.23 ± 8.95	62.50 ± 6.66	–1.295	0.197
Male,%	37 (50.7%)	31 (48.4%)	0.069	0.793
Disease duration, y	3 (1, 5)	NA	NA	NA
UPDRS III score	25 (16.5, 37.0)	NA	NA	NA
H-Y stage	2.5 (2, 3)	NA	NA	NA
LEDD, mg/day	400 (343, 591)	NA	NA	NA
MMSE score	26 (21, 29)	NA	NA	NA
PDSS score	113.0 (93.0, 123.5)	NA	NA	NA

Mean ± standard deviation or median (interquartile range). MMP3, matrix metallopeptidase 3; MMP9, matrix metallopeptidase 9; UPDRS, Unified Parkinson’s Disease Rating Scale; H-Y stage, Hoehn–Yahr stage; LEDD, levodopa equivalent daily dose; MMSE, Mini Mental State Examination; PDSS, Parkinson’s disease sleep scale; t, t-value in t-test; χ^2^, Chi-square value in chi-square test; NA, not applicable/not available.

### MMP3 and MMP9 levels in PD patients and in healthy controls

Patients were categorized according to H-Y stages in early-stage PD (*n* = 51) and advanced-stage PD (*n* = 22). Serum MMP3 levels were significantly decreased in PD patients compared with the control group [13.12 (9.40, 20.04) vs. 15.37 (11.33, 24.41) ng/ml, *P* = 0.033]. There were statistically significant differences in MMP3 levels among the three groups (early-stage PD patients, advanced-stage PD patients and healthy controls) [12.56 (9.30, 17.44) vs. 15.31 (8.96, 25.49) vs. 15.37 (11.33, 24.41) ng/ml; *P* = 0.017]. Significantly lower MMP3 levels were observed in the participants with early-stage PD than in the controls [12.56 (9.30, 17.44) vs. 15.37 (11.33, 24.41) ng/ml; *P* = 0.004]. There was no statistically significant difference in serum MMP3 levels in patients with advanced-stage PD compared to healthy controls [15,31 (8.96, 25.49) vs. 15.37 (11.33, 24.41) ng/ml; *P* = 0.350]. In addition, compared to those in PD patients with early-stage disease, MMP3 levels in advanced-stage PD patients were higher, while there were no significant differences between MMP3[12.56 (9.30, 17.44) vs. 15,31 (8.96, 25.49) ng/ml; *P* = 0.220].

Serum MMP9 levels were significantly increased in PD patients compared with the control group [522 (419, 729) vs. 329 (229, 473) ng/ml *P* < 0.001]. There were statistically significant differences in MMP9 levels among the three groups (early-stage PD patients, advanced-stage PD patients and healthy controls) [503 (390, 729) vs. 564 (504, 769) vs. 329 (229, 473) ng/ml *P* < 0.001]. Compared with the control group, MMP9 level of early-stage PD patients [503 (390, 729) vs. 329 (229, 473) ng/ml; *P* < 0.001] and MMP9 level of advanced-stage PD patients [564 (504, 769) vs. 329.13 (229, 473) ng/ml; *P* < 0.001] were significantly higher. Moreover, compared to those in PD patients with early-stage disease, MMP9 levels in advanced-stage PD patients were higher [503 (390, 729) vs. 564 (504, 769) ng/ml; *P* = 0.006] (Figure 1).

**FIGURE 1:** Serum MMP3 and MMP9 levels in PD patients and contr subjects. **(A)** MMP3 levels in the PD group with early-stage disease were highly decreased in the serum compared with the controls; There was no statistically significant difference in serum MMP3 levels in patients with advanced-stage PD compared to healthy controls; Compared to PD patients with early-stage disease, MMP3 levels in advanced-stage PD patients were higher, while there were no significant differences. **(B)** MMP9 in the PD group with early-stage disease was increased in the serum compared with the controls; Serum levels were elevated in the advanced-stage PD group relative to the control group; Compared to PD patients with early-stage disease, MMP9 levels in advanced-stage PD patients were higher. PD, Parkinson’s disease; MMP3, Matrix Metalloproteinase 3; MMP9, Matrix Metalloproteinase 9. The central line in each box indicates the median, box edges mark the first and third quartiles, and limits of the vertical lines show ranges. NS, no significance; *P < 0.05.

The diagnostic accuracy of PD patients and healthy controls was determined by ROC analysis. MMP3 (*AUC* = 0.606; *P* = 0.033, *95% CI* 0.511-0.700), at a cutoff value of 11.22 ng/ml, showed 42.47% sensitivity (Se) and 76.56% specificity (Sp). MMP9 (*AUC* = 0.780; *P* < 0.001, *95% CI* 0.703-0.857), at a cutoff value of 438.68 ng/ml, showed 74.00% Se and 74.4% Sp (Figure 2).

**FIGURE 2:** ROC curve for serum MMP3 and MMP9 levels comparing the PD group and healthy control group. ROC curve, receiver operating characteristic curve; AUC, area under the curve; CI, confidence interval.

### Correlation of serum MMP3 and MMP9 levels with disease duration and disease severity in Parkinson’s disease patients

We found that the level of serum MMP3 was positively correlated with the course of disease (*r* = 0.297, *P* = 0.011) and with the UPDRS Part III score (*r* = 0.389, *P* < 0.001). In addition, the level of serum MMP9 was positively correlated with the UPDRS Part III score (*r* = 0.279, *P* = 0.017). Serum MMP9 level was not correlated with the course of disease (*r* = 0.063, *P* = 0.594) (Figure 3). There was no significant correlation between serum MMP3 or MMP9 levels and the LEDD.

**FIGURE 3:** Correlation of serum matrix metalloproteinase 3 (MMP3) and matrix metalloproteinase 9 (MMP9) levels with disease duration and disease severity in PD patients. **(A)** Serum MMP3 levels were positively correlated with disease duration (Spearman’s correlation coefficient *r* = 0.297, *P* = 0.011, and *n* = 73). **(B)** Serum MMP3 levels were positively correlated with UPDRS part III scores (Spearman’s correlation coefficient *r* = 0.389, *P* = 0.001, and *n* = 73). **(C)** Serum MMP9 levels were positively correlated with UPDRS part III scores (Spearman’s correlation coefficient *r* = 0.279, *P* = 0.017, and *n* = 73). *P < 0.05. **(D)** Serum MMP9 level was not correlated with the course of disease (*r* = 0.063, *P* = 0.594, and *n* = 73).

### Correlation analysis of non-motor symptoms and serum MMP3 and MMP9 levels in Parkinson’s disease patients

Correlation analysis revealed that MMP3 levels were positively correlated with the NMSS total score (*r* = 0.271, *P* = 0.020) as well as the single-item scores for item six, assessing gastrointestinal problems (*r* = 0.333, *P* = 0.004). Additionally, MMP9 levels were positively correlated with the NMSS total score (*r* = 0.234, *P* = 0.047) (Table 2). We found a negative correlation between serum MMP3 levels and the PDSS score (*r* = –0.246, *P* = 0.036). In addition, serum MMP9 levels did not correlate with MMSE scores (*r* = –0.165, *P* = 0.162) (Figure 4).

**TABLE 2:** Correlation analysis of non-motor symptoms and serum MMP3 and MMP9 levels in PD patients.

	Medians (quartile ranges)	MMP3		MMP9	
			
		Spearman rank	*P*	Spearman rank	*P*
NMSS total score	40.00 (24.50, 65.00)	0.271	0.020*	0.234	0.047*
**NMSS component score**					
Cardiovascular	0.00 (0, 2)	–0.115	0.335	0.073	0.537
Sleep/fatigue	8.00 (3, 14)	0.120	0.311	0.093	0.435
Mood/cognition	7.00 (3, 14)	0.074	0.534	0.076	0.525
Perceptual Problems/hallucinations	0.00 (0, 2)	0.039	0.743	–0.012	0.920
Attention/memory	3.00 (1, 8)	0.188	0.111	0.102	0.390
Gastrointestinal tract	3.00 (1, 8)	0.333	0.004*	0.207	0.079
Urinary	4.00 (0, 12)	0.105	0.377	0.132	0.266
Sexual function	0.00 (0, 0)	–0.068	0.569	0.138	0.244
Miscellaneous	4.00 (1, 10)	0.154	0.193	0.158	0.180

NMSS, The Non-motor Symptoms Scale for Parkinson’s disease.

**FIGURE 4:** Correlation of serum Matrix Metalloproteinase 3 (MMP3) with the PDSS score and matrix metalloproteinase 9 (MMP9) levels with the MMSE score in PD patients. **(A)** Serum MMP3 levels were negatively correlated with the PDSS score (Spearman’s correlation coefficient *r* = –0.246, *P* = 0.036, and *n* = 73). *P < 0.05. **(B)** Serum MMP9 levels were negatively correlated with the MMSE scores (Spearman’s correlation coefficient *r* = –0.165, *P* = 0.162, and *n* = 73) but were not statistically significant.

Next, we evaluated differences in MMP3 and MMP9 levels between the two subgroups. 17 patients exhibited sleep disorder and 21 patients showed cognitive dysfunction. No significant differences were found in MMP3 levels according to sleep disorder or cognitive dysfunction. However, serum MMP9 levels were higher in PD patients with cognitive dysfunction compared to cognitively normal PD patients [658 (505, 877) vs. 502 (398, 608) ng/ml, *P* = 0.008].

## Discussion

Our study first found that the peripheral MMP3 level of PD patients decreased, while the MMP9 level increased. After H-Y stage classification, MMP3 levels were found to be significantly lower in early-stage PD patients than in healthy controls, while MMP9 levels were found to be significantly higher in early-stage and advanced-stage PD patients than in healthy controls. MMP3 may be passively localized with Lewy bodies and play a key role in the progression of PD (Choi et al., 2011). Cells can also capture it in inclusion bodies, which is part of the cell protection mechanism, which may be related to reducing the proliferation of toxic molecules (Arrasate et al., 2004). Therefore, MMP3 levels in postmortem brain tissue of PD patients are elevated. MMP3 released by stressed DA neurons are involved in disease progression (Kim et al., 2005, 2007). When patients with PD develop symptoms, more than 50% of the dopaminergic neurons have been damaged, and the peripheral/serum MMP3 level released by the injured neurons may decrease. The role of MMP3 *in vivo* is complex, and its mediating role in PD patients is still unclear. In an MPTP-induced PD animal model, alpha-synuclein was shown to upregulate MMP9 activity in astrocytes and microglia (Lorenzl et al., 2004), which may be related to dopamine neuronal cell death (Kim S. Y. et al., 2010). Persistent neuroinflammation induced by MMP9 is associated with progressive degeneration of the substantia nigra-striatum circuit, suggesting a role in inflammatory exacerbation (Annese et al., 2015). In addition, we found that the level of MMP9 in patients with advanced-stage PD was higher than that in patients with early-stage PD. It is believed that patients have higher levels of inflammation in late stages than in early-stage stages. The cellular sources of MMPs in the brain include infiltrating leukocytes and inherent central nervous system cells (Yong et al., 2001). MMP3 disrupts the blood–brain barrier by attacking tight junctions and basal layer proteins, which contribute to neutrophil influx into the brain (Gurney et al., 2006). MMP9 is secreted in parallel with MMP3, and labor is divided to degrade different extracellular matrices (Chin et al., 1985). MMP9 was found to be a product of neutrophils (Sopata and Dancewicz, 1974), neutrophils with potential MMP9 carry it into the brain during inflammation, and disruption of the blood–brain barrier may also increase the permeability of plasma proteins (Opdenakker et al., 2001; Sellebjerg and Sørensen, 2003). Therefore, we believe that MMP3 and MMP9 in peripheral blood may reflect changes in the central nervous system. Finally, this is a controversial area of research with many gaps to be filled.

This study shows that MMP3 levels in PD patients were significantly positively correlated with the course of disease and UPDRS III score. More than 50% of dopaminergic neurons are damaged in PD patients, there may be a neuronal compensatory situation, and the compensatory capacity gradually increases with the duration of the disease. This suggesting that decreased serum MMP3 levels may play an important role in PD. In addition, we found a positive correlation between serum MMP9 levels and UPDRS III score, which may be related to the state of inflammation in the progression of PD (Annese et al., 2015). The sensitivity and specificity of serum MMP9 levels show that it can be used to distinguish PD patients from the control group, providing a basis for the diagnosis of PD. AUC values based on serum MMP3 levels are of limited value to provide a basis for the diagnosis of PD.

The characteristics of PD are not merely movement disorders; the prevalence and importance of many non-motor symptoms, including gastrointestinal dysfunction, sleep disorders, bladder dysfunction, and even fatigue, are increasingly being recognized (Pfeiffer, 2016). Subsequently, we analyzed the correlation of MMP3 and MMP9 levels in PD patients with NMSS alone. We found that serum MMP3 levels in PD patients were mainly related to the Item 6 gastrointestinal score. Among gastrointestinal dysfunctions such as salivation, dysphagia, gastroparesis, and constipation, constipation is the most common non-motor symptom of PD (Pfeiffer, 2003). Previous studies have shown significant differences in brain activity and functional connectivity between PD patients with and without constipation (Zheng et al., 2022). We found that the occurrence of gastrointestinal problems in PD patients was related to the level of MMP3. MMPs, by degrading the lamina propria matrix, are the main pathway by which T cells cause intestinal injury (Pender et al., 1997). MMP3 is upregulated in the intestine in inflammatory bowel disease and may play an important role in tissue remodeling and destruction (Heuschkel et al., 2000; Von Lampe et al., 2000; Gordon et al., 2008).

Sleep-wake abnormalities occur in disorders with impaired DA release, and inPD, up to 90% of patients suffer from some form of dyssomnia (Kurtis et al., 2013; Radwan et al., 2019). Sleep disturbance is related to the evolution of PD itself and may be related to the destruction of dopaminergic homeostasis (Barraud et al., 2009). Dopamine is produced mainly in the substantia nigra (SN) and ventral tegmental area (VTA) in the brain. VTA dopaminergic neurons produce and maintain arousal (Eban-Rothschild et al., 2016). Additionally, DA regulates the circadian rhythm through the suprachiasmatic nucleus (SCN) (Grippo et al., 2017), and DA in the substantia nigra pars compacta promotes sleep (Qiu et al., 2016). PD patients have varying degrees of damage to both substantia nigra and ventral tegmental dopaminergic neurons (Geibl et al., 2019), and MMP3 has also been associated with dopamine loss in PD patients. After subgroup analysis, sleep disorders were higher than non-sleep disorders, but the difference was not significant, which may be related to the different levels of MMP3 compensation in advanced-stage PD patients. This may explain the correlation between MMP3 levels and sleep disorders in PD patients.

We found significant differences in MMP9 levels between the cognitive impairment subgroups and cognitive integrity subgroups. Therefore, we suggest that the occurrence of cognitive impairment in PD patients is associated with elevated levels of MMP9. Cognitive dysfunction is common in PD patients, and it usually affects memory, attention and execution, as well as visuospatial ability (Aarsland et al., 2010). Several studies have demonstrated the damaging effects of MMP9 on cognition and memory. Previous studies have shown that MMP9 activity in brain samples from patients with mild cognitive impairment is significantly higher than that in patients with normal cognitive function and that MMP9 activity is negatively correlated with the MMSE score (Bruno et al., 2009). Elevated peripheral MMP9 levels may increase neurodegeneration and cognitive decline (Abe et al., 2020). The long-term potentiation (LTP) maintenance mechanism induced in slices of MMP9 overexpressing rats almost disappears, and MMP9 overexpression can damage LTP (Wiera et al., 2013). Based on these findings, we can infer that the increase in MMP9 levels may be one of the causes of the related learning and memory defects.

There are several limitations of this study. First, whether peripheral MMP3 and MMP9 levels reflect central substance activity is still controversial. Second, it is necessary to explore the relationship of the disorder of regulatory balance between MMPs and tissue inhibitors of metalloproteinases (TIMPs) with the pathogenesis of the disease. Third, this was a cross-sectional study. Therefore, longitudinal studies are needed to clarify the relationships between the development of PD and serum MMPs levels in the presence of various confounding factors.

## Conclusion

This study found for the first time that the level of MMP3 was decreased, and the level of MMP9 was increased in PD patients. At the same time, a potential association was found between serum MMP3 and MMP9 levels and non-motor symptoms in PD patients. The levels of MMP3 and MMP9 can be used to evaluate sleep disorders and cognitive function in PD patients, respectively.

## Data availability statement

The original contributions presented in this study are included in the article/supplementary material, further inquiries can be directed to the corresponding author.

## Ethics statement

The studies involving human participants were reviewed and approved by Ethics Committee of Henan Provincial People’s Hospital. The patients/participants provided their written informed consent to participate in this study.

## Author contributions

CL, JM, and HY completed the topic selection and study design. CL conducted the experiments. DG, LD, QC, and KL conducted the literature search, acquisition of data, and study supervision. XL, DY, YF, QG, SC, and DL performed the statistical analysis and interpretation of data. CL and JM drafted the manuscript. All authors contributed to the manuscript and gave final approval.
